The article "Effect of CICARE Communication Mode on Disease Uncertainty, Self-Nursing Ability, and Quality of Life in Patients with Coronary Atherosclerotic Heart Disease after Percutaneous Coronary Intervention" was retracted in 2023. Reasons: unreliable results or conclusions; concerns about the data; concerns about the peer review; concerns about the citations.

# Effect of CICARE Communication Mode on Disease Uncertainty, Self-Nursing Ability, and Quality of Life in Patients with Coronary Atherosclerotic Heart Disease after Percutaneous Coronary Intervention

**DOI:** 10.1155/2022/8654449

**Published:** 2022-08-05

**Authors:** Hui Hu, Ayong Zhang, Zhen Wang

**Affiliations:** Operating Room, Wuhan Asian Heart Hospital, 430022, China

## Abstract

**Objective:**

To study the effect of CICARE (Connect, Introduce, Communicate, Ask, Respond, Exit) communication mode on disease uncertainty, self-nursing ability, and quality of life in patients with coronary atherosclerotic heart disease (CAD) after percutaneous coronary intervention (PCI).

**Methods:**

From January 2021 to December 2021, 102 patients with CAD after PCI were randomly divided into a research group (*n* =51) and a control group (*n* =51). The former received CICARE communication model nursing intervention, and the latter received routine doctor-patient communication nursing. To study the scores of disease uncertainty scale (MUIS), Frankl treatment compliance scale (Frankl), self-care ability scale (exercise of self-care-a), quality of life scale (WHOQOL-BREF), and Newcastle nursing satisfaction scale (NSNS) before and 1 week after nursing.

**Results:**

After one week of nursing, the MUIS score of the research group was lower than that of the control group, and the score of Frankl treatment compliance scale of the research group was higher than that of the control group. After 1 week of nursing, the ESCA score of the research group was higher compared to the control group (*p* < 0.05), and the WHOQOL-BREF score of the research group was higher compared to the control group (*p* < 0.05). After one week of nursing, the NSNS score of the research group was higher compared to the control group (*p* < 0.05).

**Conclusion:**

The application value of CICARE communication mode nursing intervention in patients with CAD after PCI is more remarkable, and it is more helpful to reduce patients' disease uncertainty, enhance treatment compliance, promote patients' self-nursing ability, and strengthen quality of life and nursing satisfaction.

## 1. Introduction

Coronary atherosclerotic heart disease (CAD) is a kind of heart disease caused by coronary artery atherosclerosis, which leads to vascular stenosis, obstruction, myocardial ischemia, hypoxia, or necrosis, referred to as CAD [1, 2]. According to the statistics of the World Health Organization, 17.9 million people die of various cardiovascular diseases every year, of which about 7.4 million die of CAD [3]. In recent years, with the enhancement of China's economy, the change of people's lifestyle, and the arrival of an aging society, the incidence of coronary atherosclerotic heart disease is increasing year by year. According to statistics, there are 330 million patients with cardiovascular disease in China, of which 11 million are coronary atherosclerotic heart disease, accounting for more than 40% of the deaths of residents. The number of patients discharged from cardiovascular disease is increasing, and the total cost of hospitalization for cardiovascular disease is also increasing. Data indicates that in 2016, the total hospitalization cost of acute myocardial infarction in China was 19.085 billion yuan, and the average hospitalization cost was 26056.9 yuan, with an average annual growth rate of 7.12% [4]. The disease burden of CAD in China is increasing day by day, which has become a major public health problem. In order to reduce the family and social burden and prevent and cure CAD, it is urgent to enhance the level of treatment and rehabilitation of CAD. We should also pay attention to popularizing health knowledge.

At present, one of the main treatment methods of CAD is percutaneous coronary angioplasty (PCI), that is, percutaneous coronary intervention, which refers to the transcatheter and stent with balloon dilator sent to the narrow coronary artery through the femoral artery or radial artery, in order to dredge the narrow or blocked coronary artery lumen and then enhance myocardial blood perfusion [5]. Studies have indicated that PCI has the characteristics of less trauma, short operation time, and rapid recovery, which can effectively reduce the mortality of patients and is currently recognized as one of the effective means of revascularization when treating CAD [6, 7]. However, although many clinical trials have confirmed the effectiveness of PCI in the treatment of coronary atherosclerotic heart disease, PCI also has some limitations. Restenosis after PCI seriously affects clinical benefits. Up to 30% of patients developed restenosis within 6 months after operation. Even if drug-eluting stents (DES) are widely used, the restenosis rate is still 10% [8]. The long-term effect of PCI is affected by in-stent restenosis and coronary microcirculation disturbance [9, 10]. From the point of view of the new medical model, interventional therapy is still a palliative treatment, which can mechanically recanalize blood vessels, but it cannot reverse or delay the biological process of atherosclerosis. CAD is a disease caused by many factors. Patients still need to adhere to long-term medication and regular reexamination and maintain good living habits after discharge, which brings a lot of restrictions to patients' life, which makes it difficult for patients to adapt to life after illness and poor self-care ability. It leads to the decrease of the quality of life [11]. How to take effective means of doctor-patient communication to enhance patients' awareness of their own condition is of great significance to promote disease symptoms and reduce the occurrence of complications, which should be concerned by clinical workers.

As we all know, good nurse-patient communication can improve the recovery rate of patients to a great extent, but communication barriers seriously affect the nurse-patient relationship, and even bring disputes, resulting in tragic consequences [12]. With poor communication, medical staff cannot get disease and treatment-related information from patients, indirectly leading to the occurrence of adverse events. In the study of nurse-patient communication, some scholars pay more attention to psychological communication and health education. Only by adopting scientific communication methods and requiring nurses to master more communication methods can we promote the actual communication effect between them and patients. CICARE communication mode includes six steps: Connect (contact), Introduce (introduction), Communicate (communication), Ask (ask), Respond (answer), and Exit (leave). It is a process-oriented communication mode adopted by American medical institutions, which is mainly adopted in face-to-face communication between doctors and patients. After research, relevant researchers have found that under the clear guidance of this step, patients' satisfaction with health care is showing a remarkable upward trend [13]. Therefore, this study enrolled 102 patients with CAD after PCI in our hospital from January 2021 to December 2021 to explore the influence of CICARE (Connect, Introduce, Communicate, Ask, Respond, Exit) communication mode on disease uncertainty, self-nursing ability and quality of life of patients after percutaneous coronary intervention (PCI). The report is as follows.

## 2. Patients and Methods

### 2.1. General Information

From January 2021 to December 2021, 102 patients with coronary atherosclerotic heart disease after PCI were randomly divided into research group (*n* =51) and control group (*n* =51). In the control group, the age ranged from 54 to 73 years, with an average of (60.42 ± 3.63) years, including 33 males and 18 females; in the research group, the age was 55 to 75 years old, with an average of (60.96 ± 3.58) years old, including 31 males and 20 females. There exhibited no statistical significance in the general data. This study was permitted by the Medical Ethics Association of our hospital, and all patients signed informed consent.

Inclusion criteria: (1) in accordance with the diagnostic criteria of CAD [14], confirmed by coronary angiography and treated with PCI; (2) 18-75 years old; (3) within 1-3 months after PCI; (4) signed informed consent and voluntarily participated in this study. Exclusion criteria: (1) patients with cognitive impairment or history of mental illness; (2) patients with other serious chronic diseases, such as malignant tumor, severe heart, brain, kidney, and other diseases.

### 2.2. Treatment Methods

#### 2.2.1. Technical Route

Technical route is indicated in Figure 1.

#### 2.2.2. Intervention Scheme

Control group: Routine doctor-patient communication nursing. That is, to guide perioperative matters needing attention, medication guidance, and discharge matters needing attention. The scheme of the research group: the research group adopted CICARE communication mode for nursing intervention. The main results are as follows: (1) set up a nursing intervention group with CICARE communication mode. Establish nursing manual based on CICARE communication mode: make nursing manual based on CICARE communication mode according to literature review and the content of transfer health education in the hospital where this research project is located; (2) to carry out nursing intervention training of CICARE communication mode. The training time is on Tuesday and Thursday afternoons every week, and the training content is the same twice a week. Nurses can choose the training time according to their own time and ensure to attend the training once or twice a week. Carry on the training and examination by the way of situational exercise, pay attention to the tone, manner, appearance, and body language in the course of the examination, and each responsible nurse needs to pass the examination; (3) to implement nursing intervention based on CICARE communication mode: 1) C-contact nursing. We should keep smiling and make contact with each other with reasonable address each time, so as to make patients feel intimacy and trust and establish a good foundation of trust with their families. 2) I-introduce nursing. Take the initiative to introduce to the patients the location of the ward, the mode of arrival and environment, the working time of the ward and the system of accompanying visits, the nursing mode of the ward, and the situation of the medical staff, so that the family members of the patients can understand the situation of the general ward in advance and eliminate the strangeness and tension of the patients to the medical environment. 3) C-communication nursing. Adopt one-to-one health education service, communicate well with patients, introduce the clinical medical knowledge of CAD and PCI, and advise postoperative precautions to make patients rest assured. Help to eliminate the patient's inner sense of stress, disease uncertainty, let them relax. Be fully aware of the adverse effects of bad emotions on patients' compliance, symptom improvement, and disease control. Actively pay attention to the psychological changes of patients, and assess the severity, patiently guide patients to talk, can treat patients as relatives, and give encouragement and spiritual support. 4) A-inquire about nursing care. Evaluate the patient's current awareness, activities, self-care ability and channel, and diet, so that the patient's family members understand the basic situation of the patient, what kind of care and rehabilitation difficulties may exist. 5) R-answer. In view of the patients' questions, we should answer them actively and patiently, eliminate the patients' sense of disease uncertainty, avoid negative emotions affecting the PCI operation, and write down the points for attention of the patients' family members to assist in taking care of the patients according to the patient's condition. 6) E-leave nursing. Inform the patients' family members of the traffic next to the hospital, medical expenses inquiry, medical insurance payment methods, the use of other medical resources, and other warm tips, and inform the family members of information manuals such as other ways to solve the problem.

### 2.3. Observation Index

1. The Mishel uncertainty in illness scale (MUIS) scores before nursing and one week after nursing were studied. The MUIS scale has a total of 32 items, using the Likert 5 scale (1 point to 5 points) scoring method, with a total score range of 32 to 160 points [15]. The higher the score, the stronger the uncertainty of the disease
2. The scores of Frankl treatment compliance scale were compared before and after one week of nursing. The score of Frankl Compliance scale is as follows: 1: refusal, pain; 2: uncooperation, reluctance; 3: use, indifference; 4: active cooperation, enjoyment [16]. Higher scores represent better compliance
3. The self-care ability measurement scale (ESCA) scores before and after 1 week of nursing in the two groups were studied. The ESCA scale includes 43 items in 4 evaluation items, including self-concept (8 items), self-care responsibility (6 items), self-care skills (12 items), and health knowledge level (17 items) [17]. Scored on a 5-point scale from 0 to 4, of which 4: very similar to me; 3: somewhat like me; 2: not sure; 1: somewhat not like me; 0: very similar I. The total score is 172 points. The higher the score, the stronger the self-care ability
4. The short form for measuring quality of life (WHOQOL-BREF) before nursing and after 1 week of nursing. The WHOQOL-BREF scale includes a total of 26 items, including four areas: physiology, psychology, social relations, and environment [18]. Each item is scored from light to heavy, and 3 items need to be counted in reverse. The score of each field = the average score of the field X4; the higher the field score, the better the quality of life in the corresponding field
5. The Newcastle Satisfaction with nursing scales (NSNS) scores before and after 1 week of nursing were studied. The NSNS scale has a total of 19 test items, and each item is evaluated on a 5-point scale from 1 to 5, of which 1: means very dissatisfied; 2: means dissatisfied; 3: means Generally satisfied; 4 points: satisfied; 5 points: very satisfied [19]. The higher the score, the higher the satisfaction

### 2.4. Statistical Analysis

The statistical analysis of the data in this study uses SPSS24.0 software, and the statistical graphics are drawn by GraphPad Prism8.0. The measurement data with normal distribution were presented by mean ± standard deviation ($\overset{-}{x}\pm S$). Paired sample *t*-test was used for intra-group comparison, and independent sample *t*-test was used for inter-group comparison. *p* < 0.05 exhibited statistically remarkable. If it is not consistent, it is presented by the median (lower quartile to upper quartile). Paired sample nonparametric test is employed for intra-group comparison, and independent sample nonparametric test is adopted for inter-group comparison. The grade data were examined by FISHER accurate method; *p* < 0.05 indicated there exhibited statistical significance.

## 3. Results

### 3.1. To Study the Scores of MUIS Scale before Nursing and 1 Week after Nursing

Before nursing, there exhibited no remarkable difference in MUIS score (*p* > 0.05); after one week of nursing, the MUIS score of the research group was lower (*p* < 0.05). This result indicates the research group is better than the control group, as indicated in Table 1.

### 3.2. To Study the Scores of Frankl Treatment Compliance Scale before Nursing and 1 Week after Nursing

Before nursing, there exhibited no remarkable difference in the scores of Frankl treatment compliance scale (*p* > 0.05); after one week of nursing, the score of Frankl treatment compliance scale in the research group was higher (*p* < 0.05); this result indicates the research group is better than the control group. as indicated in Table 2.

### 3.3. To Study the Scores of ESCA Scale before Nursing and 1 Week after Nursing

Before nursing, there exhibited no remarkable difference in ESCA score (*p* > 0.05); after one week of nursing, the ESCA score of the research group was higher (*p* < 0.05), this result indicates the research group is better than the control group, as indicated in Table 3.

### 3.4. To Study the WHOQOL-BREF Score before Nursing and One Week after Nursing

Before nursing, there exhibited no remarkable difference in WHOQOL-BREF score (*p* > 0.05); after one week of nursing, the WHOQOL-BREF score of the research group was higher (*p* < 0.05); this result indicates the research group is better than the control group, as indicated in Tables 4–7.

### 3.5. The NSNS Scores Were Observed before Nursing and 1 Week after Nursing

Before nursing, there exhibited no statistical difference in NSNS scores (*p* > 0.05); after one week of nursing, the NSNS score of the research group was higher (*p* < 0.05). This result indicates the research group is better than the control group, as indicated in Table 8.

## 4. Discussion

Since 1977, the first case of percutaneous transluminal coronary angioplasty (PTCA) has been adopted in clinic, which indicates that the treatment of CAD has entered the era of interventional technology [20]. PCI has gradually matured and popularized and developed rapidly. According to the statistics of the National Center for Quality Control of Cardiovascular Diseases, the total number of PCI cases in China in 2018 was 915256, ranking first in the world [21]. Clinical studies have shown that although interventional therapy can effectively help patients treat diseases and alleviate coronary artery stenosis, there is still a risk of restenosis if improper nursing [22–25]. Patients with CAD after PCI cannot adjust the physical and mental stress caused by disease in time during the long-term struggle with multiple diseases, worry about stent condition and fear of cardiovascular events, not only need to take cardiovascular drugs, quit smoking and alcohol, control diet, control weight, proper exercise, regular review, but also face threats such as job changes, life changes, and economic stress [26]. The uncertainty of the disease and poor compliance may bring about in-stent restenosis, which requires interventional therapy again, which increases the economic and psychological burden of patients and needs clinical attention [27].

At present, the traditional method of relying solely on nursing technology to judge the quality of nursing service is no longer suitable for the current hospital nursing work nor can it really meet the requirements of the current medical environment [28]. Under the conventional nursing mode of doctor-patient communication, medical staff simply tell the matters needing attention, the contact and communication with patients is not ideal, and they are not aware of the improvement of nursing service quality. Patients' cognitive and psychological nursing needs cannot be met and lack of cognition, which will have a certain impact on the effect of PCI surgery to a large extent, resulting in poor compliance and satisfaction of patients [29]. In clinical research, many researchers have found that nursing technology is not the main cause of tension in nurse-patient relationship, and improper words or related body movements of nursing staff may be the most direct factor leading to conflict in nurse-patient relationship [30]. In recent years, many clinical staff and related scholars have conducted a relatively in-depth and extensive discussion on the issue of nurse-patient communication. They agreed that the communication of nurses should follow the communication mode of “patient-centered” and “improving patients” medical experience [31]. CICARE communication mode specifically refers to the nursing staff in the process of communication with patients and patients' families, gradually use the six steps of this model, so as to enhance nurses to gradually transform the knowledge of human theory into the result of practical application [32]. Therefore, this paper carried out a study to study the effects of CICARE communication mode on disease uncertainty, self-care ability, and quality of life in patients with coronary atherosclerotic heart disease after PCI.

The results of this study indicated that after the implementation of CICARE communication model nursing intervention, the MUIS scale score of patients was lower compared to routine doctor-patient communication nursing (*p* < 0.05); the scores of Frankl treatment compliance scale, ESCA scale, and WHOQOL-BREF scale and NSNS score were higher compared to routine doctor-patient communication and nursing (*p* < 0.05). It is proved that the application value of CICARE communication mode nursing intervention in patients with CAD after PCI is more remarkable, and it is more helpful to reduce patients' disease uncertainty, enhance treatment compliance, promote patients' self-nursing ability, and strengthen quality of life and nursing satisfaction. This is mainly because the main results are as follows: (1) CICARE communication mode not only further standardizes the nursing behavior of nurses but also gives patients the psychological experience of being respected and cared for. Through related research, Tan Li pointed out that CICARE communication mode can be regarded as a new way of communication, which can make nursing communication more streamlined and standardized, and facilitate nurses to develop good communication habits [33]. In the study of Yuan Fang, through the application of CICARE communication model in the whole process of special examination patient pick-up and delivery service, it is found that the comprehensive quality evaluation of support staff after the implementation of this model is remarkably better than that before implementation, so it is confirmed that CICARE communication mode can not only enhance the satisfaction rate of patients but also promote the comprehensive literacy of support staff [34]; (2) the attitude of the medical staff is related to the patients' understanding of the disease. After the nursing intervention of the CICARE communication mode, the careful discussion between the nursing staff and the patients can greatly reduce the tension of the patients, build a bridge of trust, obtain the cognition of the disease, reduce the uncertainty of the disease, and enhance the treatment compliance. In the study of Zhang Liqing, after applying CICARE communication mode to nursing care in orthopedic ward, it is concluded that this model can make nurses quickly understand the needs of patients, change the new passive guidance mode of patients in the past, and effectively enhance their treatment compliance [35]. The above conclusions are further confirmed in the study of Zhang Yan and others [36]. They randomly recruited 182 inpatients and assigned them to the control group and communication group according to different modes of communication. The former group was given general communication mode, and the latter group was given CICARE communication mode. The results show that CICARE communication mode can not only effectively improve the satisfaction of patients and their families with nursing work but also avoid depression. It can be noticed that this model can greatly reduce the irritability and sadness of patients during treatment and enhance their compliance. In the study of Xie Cuiqin et al., CICARE communication mode was adopted to process and standardize the nursing work in tuberculosis ward, which proved that this communication template was very standardized and easy to implement, which not only made the whole nurse-patient communication more scientific and reasonable but also remarkably improved patients' treatment compliance [37]; (3) CICARE communication mode achieves “people-oriented.” This model can not only enhance nurses' nursing attitude and sense of responsibility but also promote communication skills, strengthen the standardization and standardization of nursing behavior, facilitate patients' condition, and enhance their quality of life, so as to enhance patients' satisfaction. Guo Linhua pointed out that the introduction of CICARE communication mode into nursing practice can clearly implement every link and let patients actively cooperate with treatment, so as to improve their self-nursing ability and quality of life, thus making patients more satisfied with nursing work [38]. Our study still has some shortcomings. Firstly, the quality of this study is limited due to the small sample size we included in the study. Secondly, this research is a single-center study and our findings are subject to some degree of bias. Therefore, our results may differ from those of large-scale multicenter studies from other academic institutes. Our research is still clinically significant and further in-depth investigations will be carried out in the future.

In conclusion, the application value of CICARE communication mode nursing intervention in patients with coronary atherosclerotic heart disease after PCI is more significant, and it is more helpful to reduce patients' disease uncertainty, enhance treatment compliance, improve patients' self-nursing ability, and strengthen quality of life and nursing satisfaction.

## Figures and Tables

**Figure 1:** Technical route.

**Table 1:** The MUIS score before nursing and after one week of nursing.

Grouping	Before nursing (points)	After 1 week of nursing (points)	*t* score	*p* value
C group (*n* =51)	67.66 ± 5.53	43.34 ± 3.28	*27.013*	*<0.01*
R group (*n* =51)	67.73 ± 5.48	38.56 ± 2.14	*35.409*	*<0.01*
*t* score	0.064	*8.716*		
*p* value	0.949	*<0.01*		

**Table 2:** The scores of Frankl treatment compliance scale before and after one week of nursing.

Grouping	Before nursing	After 1 week of nursing	*t* score	*p* value
C group (*n* =51)	1.54 ± 0.19	2.82 ± 0.11	*41.636*	*<0.01*
R group (*n* =51)	1.55 ± 0.12	3.69 ± 0.03	*123.223*	*<0.01*
*t* score	0.318	*54.492*		
*p* value	0.751	*<0.01*		

**Table 3:** The ESCA score before nursing and after one week of nursing.

Grouping	Before nursing	After 1 week of nursing	*t* score	*p* value
C group (*n* =51)	85.12 ± 5.39	118.19 ± 7.25	*26.142*	*<0.01*
R group (*n* =51)	84.14 ± 5.44	149.23 ± 8.35	*46.643*	*<0.01*
*t* score	0.904	*20.046*		
*p* value	0.363	*<0.01*		

**Table 4:** The WHOQOL-BREF-physiological scores before and after one week of nursing.

Grouping	Before nursing	After 1 week of nursing	*t* score	*p* value
C group (*n* =51)	11.29 ± 1.64	17.59 ± 2.32	*15.836*	*<0.01*
R group (*n* =51)	11.31 ± 1.65	21.36 ± 3.14	*20..234*	*<0.01*
*t* score	0.061	*6.896*		
*p* value	0.951	*<0.01*		

**Table 5:** The WHOQOL-BREF-psychological score before and after one week of nursing.

Grouping	Before nursing	After 1 week of nursing	*t* score	*p* value
C group (*n* =51)	12.11 ± 1.25	15.02 ± 2.17	*8.298*	*<0.01*
R group (*n* =51)	12.17 ± 1.39	19.58 ± 3.11	*15.534*	*<0.01*
*t* score	0.229	*8.587*		
*p* value	0.819	*<0.01*		

**Table 6:** The WHOQOL-BREF-social relations scores before and after one week of nursing.

Grouping	Before nursing	After 1 week of nursing	*t* score	*p* value
C group (*n* =51)	11.49 ± 1.12	16.71 ± 2.36	*14.270*	*<0.01*
R group (*n* =51)	11.52 ± 1.09	21.15 ± 3.25	*20.062*	*<0.01*
*t* score	0.137	*7.894*		
*p* value	0.891	*<0.01*		

**Table 7:** The WHOQOL-BREF-environmental score before and after one week of nursing.

Grouping	Before nursing	After 1 week of nursing	*t* score	*p* value
C group (*n* =51)	14.22 ± 1.13	18.01 ± 2.14	*11.184*	*<0.01*
R group (*n* =51)	14.19 ± 1.14	22.48 ± 3.33	*16.820*	*<0.01*
*t* score	0.133	*8.065*		
*p* value	0.894	*<0.01*		

**Table 8:** The NSNS scores before nursing and after one week of nursing.

Grouping	Before nursing	After 1 week of nursing	*t* score	*p* value
C group (*n* =51)	71.59 ± 5.17	82.18 ± 4.25	*11.300*	*<0.01*
R group (*n* =51)	71.63 ± 5.14	93.53 ± 2.11	*28.148*	*<0.01*
*t* score	0.039	*17.082*		
*p* value	0.969	*<0.01*		

## Data Availability

No data were used to support this study.
